The article "Comparative Effectiveness of Endoscopic Versus Pharmacological Interventions for Variceal Rebleeding in Cirrhosis: A Systematic Review" was retracted in 2025. Reasons: signs of a paper mill; unreliable results or conclusions; concerns about the authorship.

# Comparative Effectiveness of Endoscopic Versus Pharmacological Interventions for Variceal Rebleeding in Cirrhosis: A Systematic Review

**DOI:** 10.7759/cureus.72085

**Published:** 2024-10-22

**Authors:** Muath M Dabas, Muhammad Maqbool, Adees W Bedros, Hiba Mazhar, Papuna Papuashvili, Muhammad Umar, Aqsa B Bajwa, Dhruvi H Patel, Nada B Abushalha, Abid Khattak, Junaid Ahmed, Asma Mehdi

**Affiliations:** 1 Surgery, The University of Jordan, Amman, JOR; 2 Internal Medicine, Shaheed Mohtarma Benazir Bhutto Medical College Lyari, Karachi, PAK; 3 Internal Medicine, The University of Jordan, Amman, JOR; 4 Gastroenterology, Pakistan Kidney and Liver Institute, Lahore, PAK; 5 Internal Medicine, Tbilisi State Medical University, Tbilisi, GEO; 6 Internal Medicine, Faisalabad Medical University, Faisalabad, PAK; 7 Internal Medicine, Shalamar Medical and Dental College, Riyadh, SAU; 8 Internal Medicine, Civil Hospital, Surat, IND; 9 Acute Medicine, Sherwood Forest Hospitals NHS Foundation Trust, Sutton-in-Ashfield, GBR; 10 Internal Medicine, Chandka Medical College Hospital, Larkana, PAK; 11 Surgery, Rawalpindi Medical University, Rawalpindi, PAK

**Keywords:** cirrhosis, endoscopic therapy, pharmacological treatment, rebleeding prevention, variceal bleeding

## Abstract

Variceal bleeding is a critical complication in cirrhotic patients, significantly increasing morbidity and mortality risks, particularly after an initial bleeding episode. This systematic review evaluates and compares the effectiveness of endoscopic and pharmacological interventions in preventing variceal rebleeding. A comprehensive search of major databases, including PubMed, MEDLINE, Embase, the Cochrane Central Register of Controlled Trials, and Web of Science, was conducted to identify studies published within the past decade. The review focused on randomized controlled trials, clinical trials, and meta-analyses that assessed the efficacy and safety of these treatments in adult cirrhotic patients with a history of variceal bleeding. The findings suggest that endoscopic interventions, such as band ligation and early transjugular intrahepatic portosystemic shunt (TIPS) placement, effectively reduce immediate rebleeding rates and improve short-term survival, particularly in high-risk patients with advanced cirrhosis. In contrast, pharmacological strategies, including beta-blockers and vasoactive agents, provide effective long-term management with fewer adverse events, especially in patients with milder liver disease. The review underscores the importance of a personalized treatment approach that integrates both endoscopic and pharmacological therapies to optimize outcomes and reduce the burden of rebleeding. It also highlights the need for further high-quality research to clarify the long-term benefits, impact on quality of life, and cost-effectiveness of these interventions. These insights form the basis for refining clinical guidelines and improving patient-centered care in the management of variceal rebleeding.

The article "Comparative Effectiveness of Endoscopic Versus Pharmacological Interventions for Variceal Rebleeding in Cirrhosis: A Systematic Review" was retracted in 2025. Reasons: signs of a paper mill; unreliable results or conclusions; concerns about the authorship.

## Introduction and background

Variceal bleeding is a life-threatening complication in cirrhotic patients, a chronic liver condition marked by portal hypertension and variceal formation [1]. Around 40% to 95% of cirrhotic patients develop esophageal or gastric varices, with a high risk of bleeding, especially in advanced liver disease [2]. Variceal bleeding significantly increases mortality, morbidity, and healthcare costs and lowers quality of life. Current strategies to prevent variceal rebleeding combine pharmacological and endoscopic interventions, each with distinct mechanisms, efficacy profiles, and safety considerations [3].

Pharmacological treatments, such as non-selective beta-blockers and vasoactive agents, reduce portal pressure and variceal tension, lowering the risk of bleeding [4]. Endoscopic approaches, including band ligation and sclerotherapy, directly obliterate or shrink varices to reduce bleeding risk [5]. Advanced techniques like transjugular intrahepatic portosystemic shunt (TIPS) create a channel within the liver to reduce portal hypertension but may increase complications, such as hepatic encephalopathy [6].

TIPS is indicated for patients who fail standard treatments or are at high risk for rebleeding, particularly those with recurrent variceal hemorrhage or refractory ascites. While effective in reducing portal pressure, TIPS can lead to complications like hepatic encephalopathy, stent dysfunction, or infection. Endoscopic procedures, on the other hand, have contraindications such as active sepsis, uncorrected coagulopathy, or poor patient performance status. Early complications of endoscopic procedures may include perforation, infection, or aspiration, while late complications include variceal recurrence or ulceration. These factors need to be considered when determining the optimal treatment strategy for each patient. Despite these options, uncertainty remains regarding the optimal strategy to prevent rebleeding, especially given the diverse causes of cirrhosis, comorbidities, and variable treatment responses [7].

The debate on the most effective and safest intervention highlights the need for a comprehensive analysis of current evidence to guide decision-making. This systematic review synthesizes the latest findings on the comparative effectiveness of endoscopic versus pharmacological interventions in preventing variceal rebleeding, focusing on outcomes like rebleeding rates, mortality, and adverse events. By critically assessing the data, we aim to provide insights to improve patient outcomes and shape future research directions in variceal bleeding management [8].

The article "Comparative Effectiveness of Endoscopic Versus Pharmacological Interventions for Variceal Rebleeding in Cirrhosis: A Systematic Review" was retracted in 2025. Reasons: signs of a paper mill; unreliable results or conclusions; concerns about the authorship.

The main objective of this review is to evaluate and compare the effectiveness of endoscopic and pharmacological interventions in preventing variceal rebleeding in cirrhotic patients. Specifically, we address the question: "Which intervention, endoscopic or pharmacological, is more effective in reducing variceal rebleeding, mortality, and adverse events in cirrhotic patients?" This review aims to offer a nuanced understanding of the benefits and risks of each intervention type, helping clinicians optimize treatment strategies. Additionally, it identifies gaps in the literature and proposes areas for future research to enhance the quality of evidence and guide clinical practice.

## Review

Materials and methods

Search Strategy

Our search strategy was developed in line with the Preferred Reporting Items for Systematic Reviews and Meta-Analyses (PRISMA) guidelines to identify studies comparing endoscopic and pharmacological interventions for preventing variceal rebleeding in cirrhotic patients [9]. We conducted a comprehensive search across key electronic databases, including PubMed, MEDLINE, Embase, the Cochrane Central Register of Controlled Trials, and Web of Science. The search was limited to studies published between 2014 and September 2024 to ensure the inclusion of the most recent and relevant evidence.

We used a combination of keywords and Medical Subject Headings (MeSH) terms, including "cirrhosis," "variceal bleeding," "endoscopic therapy," "pharmacological treatment," and "TIPS." Boolean operators (e.g., "AND" and "OR") were employed to refine the search effectively, for example, "cirrhosis AND variceal bleeding AND (endoscopic OR pharmacological treatment)." To ensure comprehensiveness, we manually screened the reference lists of included studies and searched clinical trial registries for unpublished or ongoing studies. Only peer-reviewed articles in English were considered.

Eligibility Criteria

The eligibility criteria were carefully established to include high-quality studies that directly compared the effectiveness of endoscopic and pharmacological interventions for preventing variceal rebleeding in cirrhotic patients. We included peer-reviewed randomized controlled trials (RCTs), clinical trials, and meta-analyses that evaluated the efficacy and safety of these interventions in adult cirrhotic patients. The review focused on studies published in English over the last 10 years (January 2014 to September 2024) to ensure the use of up-to-date evidence. Only studies reporting clear outcomes on variceal rebleeding, mortality, and adverse events were included. A minimum follow-up period of six months was required to assess long-term outcomes.

The article "Comparative Effectiveness of Endoscopic Versus Pharmacological Interventions for Variceal Rebleeding in Cirrhosis: A Systematic Review" was retracted in 2025. Reasons: signs of a paper mill; unreliable results or conclusions; concerns about the authorship.

Studies were excluded if they did not directly compare endoscopic and pharmacological therapies or focused on populations with conditions other than cirrhosis, such as gastric varices or non-variceal upper gastrointestinal bleeding. We also excluded studies involving pediatric populations, animal models, or non-clinical settings to ensure relevance to adult clinical practice. Grey literature, such as conference abstracts, letters, and editorials, was excluded to prioritize rigorously peer-reviewed research. Studies lacking sufficient outcome data or with unclear methodologies were also excluded to maintain the reliability of the review.

Data Extraction

Our data extraction process was designed to ensure accuracy and consistency in the collected data for this systematic review comparing endoscopic and pharmacological interventions to prevent variceal rebleeding in cirrhotic patients. Two independent reviewers initially screened the articles based on titles and abstracts, categorizing them as "included," "excluded," or "uncertain." Articles deemed potentially relevant underwent a full-text review. We used a standardized data extraction form in Microsoft Excel (Microsoft, Redmond, WA) to systematically capture key information, including author details, year of publication, study design, sample size, intervention types, key outcomes, and limitations. Any discrepancies between the reviewers were resolved by a third reviewer to ensure the reliability of the extracted data, facilitating a thorough and objective synthesis of evidence.

Data Analysis and Synthesis

Due to the heterogeneity of study designs, populations, and intervention types, conducting a meta-analysis was deemed unsuitable for this review. Instead, we used a narrative synthesis to qualitatively assess and integrate findings from the included studies on endoscopic versus pharmacological interventions for variceal rebleeding prevention. This method allowed us to explore the effectiveness and safety of these interventions, focusing on reported outcomes such as mortality, rebleeding rates, and adverse events.

Key findings were categorized to identify overarching themes and significant variations in management strategies and outcomes. This thematic synthesis provided a clearer understanding of the comparative benefits and limitations of endoscopic and pharmacological treatments, highlighting which interventions may offer the most clinical benefit. Additionally, our synthesis identified gaps in the existing literature and inconsistencies in methodologies, offering a comprehensive overview of current research and suggesting areas for future investigation to improve outcomes in cirrhotic patients.

The article "Comparative Effectiveness of Endoscopic Versus Pharmacological Interventions for Variceal Rebleeding in Cirrhosis: A Systematic Review" was retracted in 2025. Reasons: signs of a paper mill; unreliable results or conclusions; concerns about the authorship.

Results

Study Selection Process

The study selection process for this systematic review was meticulously conducted in accordance with PRISMA guidelines to ensure the inclusion of relevant and high-quality studies. Initially, a comprehensive search across multiple electronic databases identified 203 records. Following the removal of 17 duplicate records, 186 records were screened based on titles and abstracts. Of these, 92 records were excluded for not meeting the predefined inclusion criteria. The remaining 94 reports were sought for retrieval, but 31 reports could not be retrieved. Subsequently, 63 full-text articles were assessed for eligibility. During this phase, 54 articles were excluded due to reasons such as lack of direct comparison between endoscopic and pharmacological interventions, inappropriate study populations, or insufficient outcome data. Ultimately, nine studies were included in the review, providing a robust foundation for evaluating the comparative effectiveness of endoscopic versus pharmacological interventions for preventing variceal rebleeding in cirrhotic patients. This rigorous selection process ensures that the review encompasses the most relevant and reliable evidence to address the research question effectively. The summary of the study selection process is provided in Figure 1.

**Figure 1:** The PRISMA flowchart represents the study selection process. PRISMA: Preferred Reporting Items for Systematic Reviews and Meta-Analyses

Characteristics of the Selected Studies

The study selection process for this systematic review involved a meticulous screening and evaluation of research articles to identify the most relevant studies that directly compare endoscopic and pharmacological interventions for variceal rebleeding prevention in cirrhotic patients. Out of the initial pool of records identified from multiple databases, duplicate entries were removed, and titles and abstracts were screened to exclude irrelevant studies, resulting in a more focused set of articles for further review. Full-text assessments were then conducted on the remaining studies to determine their eligibility based on predefined inclusion criteria, such as study design, population characteristics, and reported outcomes. This rigorous selection process resulted in the inclusion of nine high-quality studies comprising RCTs, meta-analyses, and network meta-analyses, which together provide a comprehensive overview of the comparative effectiveness of various treatment modalities in this patient population. The selected studies were chosen for their robust methodologies and relevance to the review's research question, ensuring that the synthesis of evidence would be both reliable and clinically applicable. The characteristics of the principle studies are given in Table 1.

The article "Comparative Effectiveness of Endoscopic Versus Pharmacological Interventions for Variceal Rebleeding in Cirrhosis: A Systematic Review" was retracted in 2025. Reasons: signs of a paper mill; unreliable results or conclusions; concerns about the authorship.

**Table 1:** Characteristics and findings of the key studies discussed in the article. RCT: randomized controlled trial; T-V: TIPS-variceal; O-S: other surgical; PPL: propranolol (beta-blocker); EVL: endoscopic variceal ligation; TFS: transplant-free survival; VH: variceal hemorrhage; TIPS: transjugular intrahepatic portosystemic shunt; HVPG: hepatic venous pressure gradient; TS: transjugular shunt; DSRS: distal splenorenal shunt; SLE: Second-look endoscopy; NSLE: no second-look endoscopy; AVB: acute variceal bleeding; HR: hazard ratio

Author	Year	Study Design	Population Size	Key Findings	Limitations	Quality Assessment	Risk of Bias
Huaringa-Marcelo et al. [10]	2021	Systematic Review and Meta-analysis	21 RCTs	No significant difference in mortality between T-V and O-S groups. T-V is associated with higher adverse events.	Moderate to low certainty of evidence. High heterogeneity in some outcomes. Only 15 studies reported adverse events.	Moderate quality; some variability in study outcomes and adverse event reporting.	Moderate risk of bias due to high heterogeneity and incomplete reporting of adverse events.
Singh et al. [11]	2022	RCT	160 (80 PPL, 80 EVL)	PPL associated with lower TFS and poor control of ascites compared to EVL. Both treatments are equally effective in preventing VH.	Small sample size, short follow-up period (12 months), lack of longer-term outcomes.	Moderate quality; small sample size and short follow-up impact strength of findings.	Moderate risk of bias due to small sample size and limited follow-up.
Lv et al. [12]	2019	RCT	129 (84 early TIPS, 45 control)	Early TIPS within 72 hours improved TFS at 6 weeks and 1 year compared to standard treatment.	Limited generalizability due to specific inclusion criteria (Child-Pugh class B or C). Possible selection bias.	High-quality, well-conducted RCT with strong methodology and sufficient follow-up.	Low risk of bias; robust randomization but some selection bias due to strict inclusion criteria.
Roccarina et al. [13]	2021	Network Meta-Analysis	66 RCTs, 6653 participants	Beta-blockers, variceal band ligation, and sclerotherapy all reduced mortality compared to no intervention.	High risk of bias across trials. Low-certainty evidence. No trials reported health-related quality of life.	Moderate quality; variability in the certainty of evidence across trials and lack of quality of life outcomes.	Moderate risk of bias due to inconsistent evidence quality and under-reporting of health-related outcomes.
Plaz Torres et al. [14]	2021	Network Meta-Analysis	48 RCTs, 3526 participants	Variceal band ligation may result in fewer serious adverse events than sclerotherapy. TIPS significantly reduced symptomatic rebleeds.	High uncertainty in many comparisons. Low to very low certainty evidence. No health-related quality of life reported.	Moderate quality; some comparisons have high uncertainty, but overall conclusions are valid.	Moderate risk of bias due to low-certainty evidence and inconsistent comparisons across trials.
Wang AJ et al. [15]	2020	RCT	252 patients	SLE significantly reduced early rebleeding and mortality compared to NSLE.	No reduction in rebleeding for secondary prophylaxis. Limited to patients with large esophageal varices. No long-term outcomes.	High quality; solid design with a large sample size and sufficient follow-up for early outcomes.	Low risk of bias; good randomization and outcome assessment, though long-term data is missing.
Simonetti RG et al. [16]	2020	Meta-Analysis	27 RCTs, 1828 participants	Very uncertain evidence on portosystemic shunts versus endoscopic interventions in reducing all-cause mortality and rebleeding.	Very low certainty of evidence due to high risk of bias, imprecision, and publication bias. Lack of quality-of-life data.	Moderate quality; affected by variability in study methodologies and outcome reporting.	Moderate risk of bias due to high imprecision and publication bias concerns.
Villanueva et al. [17]	2017	RCT	170 patients (84 HVPG-guided, 86 control)	HVPG-guided therapy significantly reduced mortality and rebleeding rates compared to standard treatment.	Study focused on patients who responded to initial therapy; results may not generalize to all cirrhotic patients. No long-term follow-up beyond 24 months.	High quality; strong randomization and well-defined patient cohort.	Low risk of bias; well-designed trial with minimal concerns over bias.
Abraldes et al. [18]	2016	RCT	158 patients (69 simvastatin, 78 placebo)	Simvastatin added to standard therapy did not reduce variceal rebleeding rates but improved survival in Child-Pugh class A/B cirrhosis.	Higher incidence of rhabdomyolysis. Composite endpoint of rebleeding and death affects clarity.	High quality; clear design and robust data on survival benefits in select patients.	Moderate risk of bias due to composite endpoint and increased side effect incidence in one group.

Discussion

This systematic review offers a comprehensive assessment of the comparative effectiveness of endoscopic versus pharmacological interventions in preventing variceal rebleeding in cirrhotic patients. The key findings suggest that both treatment modalities have distinct benefits and play specific roles in clinical practice. Endoscopic interventions, such as band ligation and sclerotherapy, were consistently effective in reducing the risk of variceal rebleeding, particularly in acute settings. Several studies demonstrated a significant reduction in early rebleeding rates and mortality associated with variceal bleeding. For instance, Wang AJ et al. highlighted the effectiveness of second-look endoscopy in significantly lowering early rebleeding rates and bleeding-associated mortality [15]. Additionally, other research indicated that early TIPS placement significantly improved short- and medium-term survival rates compared to standard treatments.

The article "Comparative Effectiveness of Endoscopic Versus Pharmacological Interventions for Variceal Rebleeding in Cirrhosis: A Systematic Review" was retracted in 2025. Reasons: signs of a paper mill; unreliable results or conclusions; concerns about the authorship.

On the other hand, pharmacological treatments, including non-selective beta-blockers and vasoactive agents, were equally effective in controlling rebleeding, particularly for long-term management. However, certain pharmacological agents, such as terlipressin and vasopressin, were linked to a higher incidence of adverse events compared to alternatives like octreotide and somatostatin, as reported by Huaringa-Marcelo et al. [10]. Additionally, studies like Abraldes et al. demonstrated that while adding pharmacological agents like simvastatin to standard therapy did not reduce rebleeding rates, it provided a survival benefit, likely due to the pleiotropic effects of statins, such as improving endothelial function, reducing portal hypertension, and attenuating inflammation [18]. These effects contribute to overall survival improvement, particularly in specific patient populations, such as those with advanced cirrhosis (Child-Pugh class A/B). These findings emphasize the need for personalized treatment strategies based on patient-specific factors, disease severity, and treatment settings to optimize outcomes in managing variceal bleeding.

The results of this review align with and expand upon existing literature regarding the management of variceal bleeding in cirrhotic patients [19]. Previous studies have debated the optimal approach for preventing rebleeding, with both endoscopic and pharmacological interventions showing varied success depending on the clinical scenario. For example, the efficacy of endoscopic band ligation in reducing rebleeding rates has been consistently supported, while pharmacological strategies like beta-blockers have been recommended for their ability to lower portal pressure, a crucial factor in variceal formation and rupture [20,21]. This review adds a deeper understanding by identifying the differential outcomes linked to specific patient subgroups and treatment settings. The benefits of early TIPS placement in patients with advanced cirrhosis and acute variceal bleeding, as shown in the studies reviewed, suggest a shift toward more aggressive interventions in high-risk populations, consistent with recent trends favoring earlier, more definitive management in acute care settings.

The article "Comparative Effectiveness of Endoscopic Versus Pharmacological Interventions for Variceal Rebleeding in Cirrhosis: A Systematic Review" was retracted in 2025. Reasons: signs of a paper mill; unreliable results or conclusions; concerns about the authorship.

Additionally, the discrepancies observed in the rates of adverse events between different pharmacological agents, such as the higher risk associated with terlipressin and vasopressin compared to octreotide and somatostatin, provide critical insights into the safety profiles of these treatments [22]. These findings are consistent with recent meta-analyses that have underscored the importance of individualized therapy, particularly in managing patients with differing levels of liver function and comorbidities [23]. The survival benefits associated with combined therapies, such as beta-blockers with endoscopic interventions, point toward a multidimensional approach to managing variceal bleeding, where the integration of multiple treatment modalities may optimize outcomes. Clinically, these insights can guide a more tailored approach to therapy, taking into account patient-specific factors such as cirrhosis severity, comorbid conditions, and bleeding history, thereby advancing the understanding and clinical management of variceal bleeding in cirrhotic patients [24]. This synthesis of evidence supports a shift toward more personalized treatment protocols that prioritize both efficacy and safety in diverse patient populations.

The observed differences in the effectiveness and safety profiles of endoscopic and pharmacological interventions for variceal bleeding in cirrhotic patients can be attributed to their distinct mechanisms of action and their interactions with the pathophysiology of cirrhosis. Endoscopic techniques, such as band ligation and sclerotherapy, directly target varices by obliterating or reducing their size, effectively preventing further bleeding. These procedures are particularly useful in acute settings where immediate control of hemorrhage is crucial, which explains the lower rates of early rebleeding observed in studies employing these methods [25]. In contrast, pharmacological agents like non-selective beta-blockers work by reducing portal hypertension through the lowering of cardiac output and promoting splanchnic vasoconstriction, which decreases pressure in the portal venous system and reduces the risk of variceal rupture. Vasoactive agents such as octreotide and somatostatin also reduce splanchnic blood flow, thereby lowering portal pressure without the systemic side effects associated with terlipressin and vasopressin, offering a safer profile [4]. The combination of these pharmacodynamic properties with the procedural benefits of endoscopic interventions suggests that a synergistic approach may be optimal for managing variceal bleeding, allowing each strategy to complement the limitations of the other. This emphasizes the importance of a tailored approach, integrating both interventions to achieve the best outcomes based on individual patient factors and clinical presentation [26].

The article "Comparative Effectiveness of Endoscopic Versus Pharmacological Interventions for Variceal Rebleeding in Cirrhosis: A Systematic Review" was retracted in 2025. Reasons: signs of a paper mill; unreliable results or conclusions; concerns about the authorship.

The primary strength of this systematic review lies in its comprehensive and methodical approach to synthesizing current evidence on the comparative effectiveness of endoscopic and pharmacological interventions in managing variceal bleeding in cirrhotic patients. The use of a robust search strategy, strict inclusion criteria, and a standardized data extraction process enhance the reliability and validity of the findings. Additionally, the narrative synthesis allowed for an in-depth exploration of the data despite the heterogeneity across studies, providing a nuanced understanding of the effectiveness and safety of treatments in various clinical contexts. However, several limitations should be acknowledged, including potential selection bias due to the exclusion of non-English studies and the reliance on published data, which may omit unpublished findings. Furthermore, the variability in study designs, patient populations, and intervention protocols posed challenges in making direct comparisons, potentially limiting the generalizability of the results. The absence of high-quality RCTs with long-term follow-up also restricts the ability to draw definitive conclusions about the long-term safety and efficacy of the interventions reviewed.

The findings of this systematic review hold significant clinical implications for the management of variceal bleeding in cirrhotic patients. The evidence supports a more individualized treatment approach, where the choice between endoscopic and pharmacological interventions should be tailored to patient-specific factors such as cirrhosis severity, comorbid conditions, and the patient’s bleeding history [27]. For instance, patients with advanced cirrhosis and a high risk of rebleeding may benefit from early and aggressive interventions like TIPS, which has been shown to improve survival outcomes in this subgroup. Conversely, patients with less severe disease or those at higher risk of complications from invasive procedures may benefit more from pharmacological management, particularly with agents like beta-blockers and octreotide, which have favorable safety profiles [28]. These findings suggest potential updates to clinical guidelines, advocating for a stratified treatment approach based on individualized risk assessments. The review also underscores the importance of regular monitoring and follow-up in managing cirrhotic patients, especially when using pharmacological strategies that require careful titration and monitoring for adverse events [29,30].

The article "Comparative Effectiveness of Endoscopic Versus Pharmacological Interventions for Variceal Rebleeding in Cirrhosis: A Systematic Review" was retracted in 2025. Reasons: signs of a paper mill; unreliable results or conclusions; concerns about the authorship.

## Conclusions

This systematic review highlights the nuanced comparative effectiveness of endoscopic versus pharmacological interventions for preventing variceal rebleeding in cirrhotic patients. The findings suggest that while endoscopic techniques like band ligation and early TIPS placement offer substantial benefits in reducing immediate rebleeding and improving short-term survival in high-risk patients, pharmacological approaches, particularly with beta-blockers and vasoactive agents, provide effective long-term management with a favorable safety profile for those with milder disease or higher procedural risk. These results underscore the need for a tailored, patient-centered approach in clinical decision-making, integrating both treatment modalities based on individual patient characteristics, cirrhosis severity, and risk factors. However, the review also identifies significant gaps in the literature, particularly regarding long-term outcomes and quality of life, underscoring the necessity for further high-quality studies to inform clinical practice and optimize treatment strategies for this complex and high-risk patient population.
